# Brain–Computer Interface–Based Communication in the Completely Locked-In State

This article has been retracted.

**DOI:** 10.1371/journal.pbio.1002593

**Published:** 2017-01-31

**Authors:** Ujwal Chaudhary, Bin Xia, Stefano Silvoni, Leonardo G. Cohen, Niels Birbaumer

**Affiliations:** 1 Institute of Medical Psychology and Behavioral Neurobiology, University of Tübingen, Tübingen, Germany; 2 Shanghai Maritime University, Shanghai, China; 3 Department of Cognitive and Clinical Neuroscience, Central Institute of Mental Health, Mannheim, Germany; 4 Human Cortical Physiology and Stroke Neurorehabilitation Section, National Institute of Neurological Disorders and Stroke, National Institutes of Health, Bethesda, Maryland, United States of America; 5 Ospedale San Camillo, IRCCS, Venice, Italy; 6 Wyss Center for Bio and Neuroengineering, Geneva, Switzerland; Rudolf Magnus Institute of Neuroscience, NETHERLANDS

## Abstract

Despite partial success, communication has remained impossible for persons suffering from complete motor paralysis but intact cognitive and emotional processing, a state called complete locked-in state (CLIS). Based on a motor learning theoretical context and on the failure of neuroelectric brain–computer interface (BCI) communication attempts in CLIS, we here report BCI communication using functional near-infrared spectroscopy (*f*NIRS) and an implicit attentional processing procedure. Four patients suffering from advanced amyotrophic lateral sclerosis (ALS)—two of them in permanent CLIS and two entering the CLIS without reliable means of communication—learned to answer personal questions with known answers and open questions all requiring a “yes” or “no” thought using frontocentral oxygenation changes measured with *f*NIRS. Three patients completed more than 46 sessions spread over several weeks, and one patient (patient W) completed 20 sessions. Online *f*NIRS classification of personal questions with known answers and open questions using linear support vector machine (SVM) resulted in an above-chance-level correct response rate over 70%. Electroencephalographic oscillations and electrooculographic signals did not exceed the chance-level threshold for correct communication despite occasional differences between the physiological signals representing a “yes” or “no” response. However, electroencephalogram (EEG) changes in the theta-frequency band correlated with inferior communication performance, probably because of decreased vigilance and attention. If replicated with ALS patients in CLIS, these positive results could indicate the first step towards abolition of complete locked-in states, at least for ALS.

## Abstract 2

"Locked in" patients suffering from advanced amyotrophic lateral sclerosis, with no reliable means of communication, can learn to answer questions requiring a “yes” or “no” thought using frontocentral oxygenation changes measurable by functional near-infrared spectroscopy.

## Author Summary

Despite scientific and technological advances, communication has remained impossible for persons suffering from complete motor paralysis but intact cognitive and emotional processing, a condition that is called completely locked-in state. Brain–computer interfaces based on neuroelectrical technology (like an electroencephalogram) have failed at providing patients in a completely locked-in state with means to communicate. Therefore, here we explored if a brain–computer interface based on functional near infrared spectroscopy (*f*NIRS)—which measures brain hemodynamic responses associated with neuronal activity—could overcome this barrier. Four patients suffering from advanced amyotrophic lateral sclerosis (ALS), two of them in permanent completely locked-in state and two entering the completely locked-in state without reliable means of communication, learned to answer personal questions with known answers and open questions requiring a “yes” or “no” by using frontocentral oxygenation changes measured with *f*NIRS. These results are, potentially, the first step towards abolition of completely locked-in states, at least for patients with ALS.

## Introduction

Communication is the process of expressing and sharing feelings, thoughts, and intentions with one another by verbal and various nonverbal means. Communication skills appear automatic but can pose severe challenges to individuals suffering from motor neuron disorders. The most devastating of motor neuron diseases is amyotrophic lateral sclerosis (ALS) [1], which is progressive and renders an individual motionless, severely affecting his or her communication ability [2]. As the disorder progresses, it destroys the respiratory and bulbar functions, forcing the individual to make vital decisions. If they opt for life and accept artificial respiration, they can no longer communicate verbally, and assistive communication devices that rely on nonverbal signals such as finger movement and gaze fixation are then used for communication [3]. In ALS, the disorder progresses in most patients until the patient loses control of the last muscular response, usually the eye muscles, a condition known as completely locked-in state (CLIS) [4].

Brain–computer interface (BCI) represents a promising strategy to establish communication with paralyzed ALS patients [5–7], as it does not need motor control. BCI research includes invasive (implantable electrodes on or in the neocortex) [8–11] and noninvasive means, including electroencephalography [12,13], functional magnetic resonance imaging (*f*MRI) [14], and functional near-infrared spectroscopy (*f*NIRS) [15], to record brain activity for conveying the user’s intent to devices such as simple word-processing programs [12]. The first BCI for communication in ALS patients with intact eye muscles was demonstrated by Birbaumer et al. (1999) [12]. With at least intact eye muscles and the rest of the body paralyzed, the condition is known as locked-in state (LIS) [4]. Since then, several invasive and noninvasive BCIs have been developed for communication in ALS patients. Noninvasive methods, namely slow cortical potential (SCP)-BCI [12,16,17], sensory motor rhythm SMR-BCI [18–20], and P300-BCI [21–24], have been utilized more frequently than invasive methods [25–27] for communication in people with ALS [6,12,27–30]. Irrespective of the types of BCI, during the BCI session patients selected letters or words after learning self-regulation of the particular brain signal or by focusing their attention to the desired letter or a letter matrix [21,23], and the attention-related brain potential selects the desired letter.

In a meta-analysis of the scientific literature of all ALS patients in CLIS [13], it was found that none of the existing techniques such as the P300 event-related brain potential (ERP), SCP, frequency analyses of various frequency bands of the electroencephalogram (EEG), and invasive electrocorticogram (ECoG) recordings [31] allowed reliable and meaningful communication with BCI. All BCI procedures mentioned above were based on effortful and explicit (conscious) voluntary control of a neuroelectric brain response such as learning with feedback and reward, during which patients learned to increase or decrease amplitudes of the SCP [12] to produce event-related desynchronization (ERD) of the central alpha-rhythm [32] to focus attention on a visually or auditorily presented sequence of letters in order to select a desired letter with the brain response. P300 [21,22,24] is also used in a similar manner to visually select a desired letter. The required activation of explicit-voluntary (controlled) attention in these BCI tasks, none of them resulting in stable learning of brain-based communication, prompted us to propose the theoretical psychophysiological notion of “extinction of goal directed cognition and thought” [13] in complete paralysis with otherwise intact cognitive processing. This theoretical account—certainly highly speculative in light of the complete lack of data about cognition and inner speech and motivational processing in CLIS—we substantiated with the failure to replicate initial positive reports about instrumental (volitional) [33,34] learning of autonomic responses in the curarized (paralysed) rat. The persistent incapability to replicate these experiments suggests that intact or partially intact motor functions and somatic-motor system mediation of autonomic functions (i.e., subtle postural or muscle tension changes to affect the desired physiological changes) is a mandatory requirement for instrumental learning and control of physiological functions. Theoretical views of this problem, like the one proposed, are not new but were expressed already in Greek philosophy by Aristotle [35] and by the philosophers of volition, particularly Arthur Schopenhauer in his monumental account of “Die Welt als Wille und Vorstellung” [36] (The World as Volition and Imagery) and during twentieth century learning theory [37,38]. Conscious of the fact that it is problematic to justify a theory on negative facts (lack of instrumental learning in the curarized rat and missing BCI control of BCIs requiring controlled attention in CLIS), we argue that [27] classical reflexive conditioning and learning might circumvent volitional effort in instrumental control. Thus, an experimental procedure involving processing of overlearned (“automatic”) questions (i.e., “Berlin is the capital of France,” “You are in pain”) asking for automatic cognitive processing only may fulfill this criterion. Thinking but not voluntary imagining affirmative “yes” and negative “no” to overlearned questions occurs effortlessly, such as automatic nodding of the head in a conversation: the extensive literature (mostly Russian) on semantic classical conditioning [39] and implicit attention and memory [40] provides ample support of this notion. However, for the case of patients in CLIS, one is faced with the dilemma that we cannot expect a learning curve characteristic of skill learning (usually exponential) or classical conditioning in a BCI task asking for overlearned “yes” and “no” responses as used on the present BCI system [29,30]. Patients were confronted in their lifetime with these questions (“Berlin is the capital of France”) before entering (or on the verge of) CLIS, and we can assume with certain confidence that no further learning at the time of assessment with the BCI is necessary and thus no learning curve can be expected. The same holds true for personal questions (“Your husband’s name is Joachim”). Thus, at an experimental level, it remains difficult to prove the speculation of intact classical conditioning but lack of instrumental voluntary learning in CLIS patients involved in a BCI task after entering CLIS. Only one patient in the literature [31] using an electrocorticographic-based BCI before and after transitioning from LIS to CLIS was published. This patient was unable to communicate with the BCI after entering CLIS. However, observation of a single case cannot serve as strong evidence comparable to the animal experiments [33,34] using curarization for the creation of reversible paralysis. We are also aware of the fact that a single case of a cognitively intact CLIS patient or curarized organism learning to instrumentally drive a BCI disproves our hypothesis. Experimental descriptions of patients with ALS or subcortical stroke in locked-in state (LIS) or who are severely paralysed using spiking frequency changes of motor neurons to move a robotic arm [10,11,41] cannot disprove our account. Patients in those studies [10,11,41] still had intact motor control of eye movements and some remaining muscles and thus could use the remaining muscular forces (somatomotor mediation) for instrumental learning and BCI control.

Because none of the BCI techniques outlined above are able to provide viable means of communication [5], the patients in CLIS due to ALS, without any muscular control, are rendered communicationless. We are then faced with the dilemma of defining communication in CLIS. Does it only mean to express one’s feelings, thoughts, and intentions in a fluent, automatized manner? Or, alternatively, does it mean to convey one’s intent or one’s feelings and thoughts to questions? As mentioned, all the existing BCIs rely on two elements: first, the neuroelectric signal (EEG or ECoG) control and second at least an intact eye muscle; the neuroelectric signal–based BCI did not work so far in patients in CLIS, in which eye movement control is lost.

A single case report by Gallegos-Ayala et al. (2014) [42] used *f*NIRS to measure and classify cortical oxygenation and deoxygenation following the “yes” or “no” thinking of the CLIS patient in response to true or false questions, respectively. The report described a CLIS patient with ALS achieving BCI control and “yes” and “no” communication to simple questions with known positive answers or negative answers and some open questions over an extensive time period. Although it was not spontaneous and voluntary, controlled communication, it at least enabled the individual without any means of communication to transmit “yes” and “no” to questions framed by family members and/or caregivers. The result opened a venue to provide at least some means of communication to individuals in CLIS who are otherwise left communicationless. Hence, an extensive study was performed on four ALS patients in CLIS to train them to communicate “yes” and “no.” In the present study, which is the first of its kind, *f*NIRS-based BCI was used for binary communication in four ALS patients in CLIS. The *f*NIRS-based BCI was employed successfully to train patients to regulate their frontocentral brain regions in response to auditorily presented questions. After training a classifier separating “yes” from “no” answers for several days, the patients were given feedback of their affirmative or negative response to questions with known answers and open questions over weeks.

## Results

The relative change in oxygenated hemoglobin (O_2_Hb) during the “true/yes” and “false/no” sentences’ interstimuli interval (ISI)—which corresponds to patients’ response interval over the frontocentral brain region of patients F, G, B, and W—are shown in Fig 1.

**Fig 1:** The averaged relative change in O_2_Hb corresponding to “yes” and “no” sentence interstimuli interval (ISI). (A) Patient F, (B) patient G, (C) patient B, and (D) patient W. (E) Channel configuration: Eight sources and eight detectors placed on the frontocentral brain region translated into 20 channels, 10 on each side of each hemisphere. For clearly displaying the relative change in O_2_Hb, 10 channels on each side of hemisphere were further subdivided in groups of 5 channels—i.e., 20 channels were divided into four groups, each consisting of 5 channels. In each subplot, the *x*-axis is time in seconds and the *y*-axis is relative change in O_2_Hb, and the five different colored lines correspond to relative change in O_2_Hb across 5 different channels, as depicted in the channel configuration map. Fig 1 data is located at https://doi.org/10.5281/zenodo.192386; https://doi.org/10.5281/zenodo.192388; https://doi.org/10.5281/zenodo.192390; https://doi.org/10.5281/zenodo.192391.

Fig 1 illustrates the change in O_2_Hb during “true/yes” sentences’ ISI—which is significantly different from the “false/no” sentences’ ISI—as corroborated by the *t*-test performed between the averages of true and false sentences’ ISI using the relative change in O_2_Hb across the four patients (*p* < 0.05), shown in Table 1, row D. The same analysis performed using the EEG signals in the time domain across all the training sessions showed no significant differences (*p* > 0.05) between the true and false sentences’ ISI across each patient, as shown in Table 1, row E. The eye movements measured with an electrooculogram (EOG) (vertical or horizontal; patients were free to use any direction) for patients F, G, B, and W while they were performing the “ja” (German word for yes) or “nein” (German word for no) thinking task showed no significant difference in the eye movements between the true and false sentences’ ISI for all patients, confirmed by the *t*-test (all *p* > 0.05), as shown in Table 1, row F, and S1B Fig.

**Table 1:** Statistics Results. Total number of (A) training, (B) feedback, and (C) open question sessions performed by each patient. The total number of sessions averaged and degrees of freedom used to perform *t*-tests between the true and false sentences’ ISI corresponding to (D) O_2_Hb, (E) EEG, and (F) EOG signals. (G) ANOVA using support vector machine (SVM) classification accuracy (CA) of O_2_Hb, EEG, and EOG signals. Post hoc *t*-test performed between (H) O_2_Hb versus EEG, (I) O_2_Hb versus EOG, and (J) EEG versus EOG classification accuracy. Note that each session contains 20 questions: 10 asking for a “yes” and 10 semantically equivalent questions asking for a “no” answer.

			Patient F	Patient G	Patient B
A) Training sessions			51	51	40
B) Feedback sessions			7	6	4
C) Open question sessions			2	2	2
D) O_2_Hb(“yes” question ISI versus “no” question ISI)	Number of sessions averaged		51	51	40
	Number of channels averaged		20	20	20
	t-value		4.01	3.96	3.67
	*p*-value		0.0001	0.0001	0.0004
E) EEG (“yes” question ISI versus “no” question ISI)	Number of sessions averaged		51	51	40
	Number of channels averaged		6	6	6
	t-value		0.97	0.61	0.83
	*p*-value		0.33	0.54	0.40
F) EOG(“yes” question ISI versus “no” question ISI)	Number of sessions averaged		51	51	40
	t-value	Horizontal EOG	.61	1.68	1.01
		Vertical EOG	.59	1.59	1.47
	*p-*value	Horizontal EOG	0.54	0.09	0.31
		Vertical EOG	0.55	0.11	0.14
G) ANOVA using classification accuracy of O_2_Hb, EEG, and EOG	F-value		20.12	7.69	16.5
	*p*-value		1.4E-08	0.0007	3.9E-08
	F-critical		3.05	3.05	3.06
H) O_2_Hb versus EEG classification accuracy	t-value		4.88	3.5	4.9
	*p*-value		1.8E-06	0.0003	2.07E-06
I) O_2_Hb versus EOG classification accuracy	t-value		5.69	4.5	5.05
	*p*-value		4.8E-08	2.5E-05	1.22E-06
J) EEG versus EOG classification accuracy	t-value		1.23	1.23	1.16
	*p*-value		0.109	0.109	0.12

Table 1 data is located at: https://doi.org/10.5281/zenodo.192386; https://doi.org/10.5281/zenodo.192388; https://doi.org/10.5281/zenodo.192390; https://doi.org/10.5281/zenodo.192391.

### ROC Curve and Classification Accuracy (CA) of O_2_Hb, EEG, and EOG Signals

The support vector machine (SVM) classifier’s classification of true sentences as true, false sentences as false, true sentences as false, and false sentences as true was used to calculate the false positive rate (FPR) and true positive rate (TPR) for each training and feedback session and also for all the training sessions and feedback sessions separately for each patient. FPR and TPR was plotted to obtain the receiver operating characteristic (ROC) curve of the binary SVM classifier during training and feedback sessions for each patient, as shown in S2 Fig, S3 Fig, S4 Fig and S5 Fig for patients F, G, B, and W, respectively. The change in oxygenated hemoglobin (O_2_Hb), EOG, and EEG power spectrum in response to true and false questions, obtained from the frontocentral region of the brain, across all the sessions from each patient was used to determine the SVM classification accuracy of "true/yes" and "false/no" answers. Successively, the daywise CA (i.e., averaging CA of all sessions in a single day) of each patient was compared to the adjusted chance-level threshold (described in BCI effectiveness metric section), as shown in Figs 2, 3, 4 and 5 for patients F, G, B, and W, respectively, and Table 2. The offline CA is reported using O_2_Hb, EEG, and EOG signals for training sessions, while online CA is reported using only O_2_Hb for feedback and open question sessions because feedback was provided online only using the O_2_Hb signal. The answering concordance between semantically paired questions ("Paris is the capital of Germany," "Paris is the capital of France"), expressed as the percentage of concordant answers over pairs' repetition, was as follows: F, 68%; G, 67%; B, 67%; W, 70%. Thus, the semantic concordance rate (SCR) ranges from 67 to 78% (see S12 Table). Median values of SCR are significantly different from 50% (all *p* < 0.0001), in which 50% is the SCR expectation of a random classifier.

**Fig 2:** Classification accuracy of Patient F. Linear SVM CA across “training sessions—offline CA” (histogram in grey), “feedback sessions—online CA” (green dot), and “open question session—online CA” (plus sign in red), obtained using (A) relative change in O_2_Hb, (B) EEG, and (C) EOG data. The classification accuracy reported here is daywise, as all the “training sessions” in a day were used to calculate the average classification accuracy of all the “training sessions” in a day. In the figure panels A, B, and C, the *x*-axis is the number of days and the *y*-axis is the classification accuracy. The solid black and dotted horizontal lines represent the chance-level threshold calculated using the metric described in the BCI effectiveness metric section for “training sessions” and “feedback sessions,” respectively. Since the feedback during the feedback and open question sessions was provided using the O_2_Hb, the online CA of the feedback and open question sessions is reported only for the *f*NIRS data. Fig 2 data is located at https://doi.org/10.5281/zenodo.191884.

**Fig 3:** Classification accuracy of Patient G. The description of this figure is the same as described in Fig 2. Fig 3 data is located at https://doi.org/10.5281/zenodo.191887.

**Fig 4:** Classification accuracy of Patient B. The description of this figure is the same as described in Fig 2. Fig 4 data is located at https://doi.org/10.5281/zenodo.191891.

**Fig 5:** Classification accuracy of Patient W. The description of this figure is the same as described in Fig 2. Fig 5 data is located at https://doi.org/10.5281/zenodo.191899.

**Table 2:** Classification statistics. **(**A) Number of days with CA above chance level; (B) number of delivered sentences with CA above chance level; (C) maximum chance-level upper limit, calculated using the metric described in BCI effectiveness metric section; and (D) mean and standard deviation of CA above chance level, obtained using the *f*NIRS, EEG, and EOG signal data for patients F, G, B, and W. For the training sessions, the CA is reported for *f*NIRS, EEG, and EOG signals. For feedback and open question sessions, CA is only reported for the *f*NIRS signal because the feedback was provided using only the *f*NIRS signal as a result of superior CA of the *f*NIRS signal during the training sessions as compared to EEG and EOG signals. Table 2 data is located at https://doi.org/10.5281/zenodo.191884; https://doi.org/10.5281/zenodo.191887; https://doi.org/10.5281/zenodo.191891; https://doi.org/10.5281/zenodo.191899.

Patient (sessions’ type)	A) Number of days with CA^1^ above chance	B) Number of sentences with CA^1^ above chance	C) Max chance-level upper limit	D) Mean CA^1^ of sessions above chance-level upper limit
	(n.^2^/tot.^3^ = %^4^)	(n.^5^/tot.^6^ = %^7^)	(%^8^)	(mean%^9^ ± std%^10^)
***f*NIRS classification accuracy**				
**F** (training)	11/14 = 78.6	929/1,020 = 91.1	64.8	69.5 ± 4.4
**F** (FB* & OQ++)	3/4 = 75.0	120/200 = 60.0	70.0	78.6 ± 6.9
**G** (training)	14/17 = 82.3	703/1,020 = 68.9	64.8	69.4 ± 4.2
**G** (FB* & OQ++)	4/5 = 80.0	80/160 = 50.0	70.0	78.8 ± 8.5
**B** (training)	9/12 = 75.0	630/800 = 78.7	64.8	69.6 ± 5.6
**B** (FB* & OQ++)	2/2 = 100.0	120/120 = 100.0	70.0	75.8 ± 6.6
**W** (training)	5/6 = 83.3	256/320 = 80.1	64.8	72.3 ± 4.3
**W** (FB*)	1/3 = 33.3	20/80 = 25.0	70.0	70.0 ± 0.0
**EEG classification accuracy**				
**F** (training)	7/14 = 50.0	546/1,020 = 53.5	64.8	65.7 ± 2.9
**G** (training)	6/17 = 35.3	555/1,020 = 54.4	64.8	66.0 ± 3.5
**B** (training)	2/12 = 16.7	44/800 = 5.5	64.8	67.5 ± 0.0
**W** (training)	4/6 = 66.7	254/320 = 79.5	64.8	68.9 ± 5.3
**EOG classification accuracy**				
**F** (training)	5/14 = 35.7	491/1,020 = 48.1	64.8	64.3 ± 2.6
**G** (training)	12/17 = 70.6	722/1,020 = 70.8	64.8	69.9 ± 5.5
**B** (training)	3/12 = 25.0	226/800 = 28.3	64.8	65.4 ± 1.9
**W** (training)	5/6 = 83.3	299/320 = 93.4	64.8	70.1 ± 4.3

^1^Classification accuracy.

^2^Number of days with *f*NIRS classification accuracy above chance-level threshold.

^3^Total number of days in which training or feedback and open question sessions were performed.

^4^Percentage of days for which *f*NIRS classification accuracy was above chance-level threshold.

^5^Number of delivered sentences with *f*NIRS classification accuracy above chance-level threshold.

^6^Total number of sentences delivered during training or feedback and open question sessions.

^7^Percentage of sentences for which *f*NIRS classification accuracy was above chance-level threshold.

^8^Maximum chance level threshold (or chance-level upper limit).

^9^Mean *f*NIRS classification accuracy of sessions above chance-level threshold.

^10^*f*NIRS classification accuracy standard deviation of sessions above chance-level threshold.

*FB: Feedback session during which participant received feedback for known questions.

++OQ: Open question session during which participant received feedback for open questions.

The results of ANOVA and post hoc *t*-test (see Table 1, row G, H, I, and J) further emphasize a significant difference between the classification accuracy of O_2_Hb versus EEG and O_2_Hb versus EOG, with no significant difference between EEG and EOG. There is one exception in the case of patient W, as no significant difference was found between the classification accuracy of O_2_Hb versus EOG. Patient W (23 y of age) suffering from juvenile ALS with an extremely rapid disease progression (2 y from diagnosis to CLIS) was not asked open questions because of the supposedly difficult emotional state at that early stage of BCI communication but continues to train the BCI at present.

### EEG Daywise Frequency Bands Analysis

The patients showed the following stable dominant frequencies: F, 6.75 Hz; G, 6.25 Hz; B, 7 Hz; and W, 8 Hz. Power spectrum density of electroencephalographic signals corresponding to "true/yes" and "false/no" sentences’ ISI acquired from channel FC6 is shown in S1 Fig. The middle-frequency bands’ (high-theta, low-alpha, and high-alpha) mean power comparison between "true/yes" and "false/no" sentences’ ISI revealed no main effects of conditions and channels in any patient (all *p* > 0.05). The middle-frequency bands’ (high-theta, low-alpha, and high-alpha) spectral features comparison between sentence presentation interval and sentences’ ISI revealed some main effects of the intervals factor, as reported in S1 Table, section A. In two (G and B) out of four patients, a smaller low-alpha band “power variability” in the sentences’ ISI compared to the sentence presentation interval was found (*p* < 0.05). In patient W, a higher high-theta, low-alpha, and high-alpha bands’ mean power in the sentences’ ISI compared to the sentence presentation interval was found (ISI was synchronized compared to sentence presentation). Patient F did not show any significant difference in the middle-frequency bands’ mean power and “power variability” (all *p* > 0.05). See Results section of S1 Text for details.

### Slow EEG Rhythms’ Relationship with *f*NIRS Classification Accuracy

The correlation analysis between *f*NIRS classification accuracy and low-frequency bands’ (those more related to vigilance) mean power revealed some interesting results (see S1 Table, section B). In three (G, B, and W) out of four patients, the median of the negative averaged correlation between low-theta band mean power and *f*NIRS classification accuracy was significantly different from zero (patient G: *r* = –0.365; patient B: *r* = *–*0.264; patient W: *r* = –0.386; all *p* < 0.05). However, in patient F, who had the longest time period in CLIS, the median of the positive averaged correlation between delta and high-theta band mean power and *f*NIRS classification accuracy was significantly different from zero (delta: *r* = 0.233; high-theta: *r* = 0.213; all *p* < 0.05). The low-frequency bands’ mean power distribution medians of successful and unsuccessful days (i.e., days with classification accuracy above chance-level threshold were considered successful) was further investigated for each patient to ascertain the difference, if any. In patient G, the low-theta band mean power of successful days was significantly smaller than that of unsuccessful days (*p* < 0.05). In patient B, the high-theta band mean power of successful days was significantly smaller than that of unsuccessful days (*p* < 0.05). This strengthens the above results of lower-frequency bands’ dominance for more unsuccessful performance. Additional details are provided in the Results section of S1 Text and in S1 Table.

## Discussion

Four patients in CLIS communicated with frontocentral cortical oxygenation-based BCI with an above-chance-level correct response rate over 70% during a period of several weeks. The performance of the binary SVM classifier across all the patients, except a few training sessions of patient B, was above chance level. None of the sessions were eliminated in the analysis, and only very few sessions had to be interrupted because of life-saving measures such as sucking saliva; thus, no bias for selecting “successful” sessions incriminates the results. Correct response rate for feedback and open questions sessions, as judged by the criteria mentioned in the Material and Methods section (Experimental Procedures), exceeded 75% in three out of four patients (F: 78.6%; G: 78.8%; B: 75.8%). Patients F, G, and B answered open questions containing quality of life estimation repeatedly with a “yes” response, indicating a positive attitude towards the present situation and towards life in general, as reported in larger samples of ALS patients [43,44]. Repeated presentation of an open question is necessary to ascertain the validity of the answer. From the ROC curve of each patient, it can be deduced that if the patient answers a question seven out of ten times with the same answer, then we can be sufficiently certain of the answer if the questioning is repeated over a long time period as done here. Correct classification of “yes” and “no” answers given mentally through *f*NIRS exceeded classification of EEG oscillations from 0–30 Hz and vertical and horizontal EOG classification. However, despite the absence of reliable eye communication in all patients as the inclusion criteria in the study and by the definition of CLIS condition, EOG classification was at some sessions, albeit rarely, above chance, mainly in patient W. Nonetheless, the inability of the social environment to perceive them and their instability and the eye tracker’s failure to use them for communication [45] prevents the use of this physiological signal.

The unreliable discrimination between "true/yes" and "false/no" sentences’ ISI by means of EEG signals (see Results section of S1 Text for details) is consistent with the results of a very similar auditory paradigm used for discriminating delayed, conditioned brain responses and tested in fourteen healthy participants [46]. However, with the exception of patient F, the comparison of middle-frequency bands’ spectral features (averaged across days) between sentence presentation interval and sentences’ ISI confirms the fact that two different states of arousal were present during sentence presentation and sentences’ ISI (see Results section of S1 Text for details). We cannot infer about the “qualia” of the two specific brain states occurring during listening to “yes–no” questions and executing the answers mentally, but at least we can state that the two mental states were different, meaning that differential cognitive processing occurred during the BCI task [47,48]. We do not have a physiologically plausible explanation as to why *f*NIRS responses to “yes” and “no” are different, as they are in three patients showing oxygenation increase during the answering interval (ISI) for “yes” responses with negligible topographical differences and oxygenation decrease during negative answers, again without topographical differences throughout the frontal cortical area. Only the very young patient W, with an extremely rapid course of the disease and a strong genetic variant, shows a variable *f*NIRS pattern with different slow oscillatory oxygenation changes between “yes” and “no” answering periods. In an animal study with nonhuman primates [49], we identified oxygenation increase as highly correlated with nearby recorded multiunit activity. Assuming a similar situation in the human brain, a “yes” answer may indicate a more coherent and more active brain state, probably supporting cellular associative binding [50–52] more readily than negative answering states. However, such a generalization remains highly speculative.

### BCI Performance and Attention-Vigilance

Three patients (G, B, and W) showed a negative averaged correlation between low-theta band mean power and *f*NIRS classification accuracy [53], meaning the smaller the low-theta band mean power, the higher the performance, except in patient F, who has been in CLIS for more than 4 y. The correlations analysis between daywise classified BCI performance and low-frequency bands across all intervals and all electrodes for each patient separately gave consistent and highly significant results (see Results section of S1 Text for details). The binary communication performance worsened with lower frequencies in two patients (G and B) as predicted. The number of days for patient W was limited (i.e., 6 d), thus it is quite unlikely to expect a significant difference in low-frequency bands’ mean power for successful and unsuccessful days (see S1 Table, section B). Decrease in vigilance reflected in slow frequencies impedes BCI performance and communication. Patient F, who had an extremely long history of CLIS without any communication over the years, showed a positive correlation in the delta and high-theta band with performance. She was the patient with very slow dominant frequency during rest, and it may be speculated that in such a deprived brain, superposition of delta and high-theta frequency represent a sign of increased attention and focus. For instance, low-theta band mean power can be used in future BCIs to stop a BCI session or to avoid the presentation of the sentences and/or questions during decreased vigilance.

For a robust validation of the BCI binary communication system in CLIS, two main unsolved questions remain: (i) the physiological identification of the cognitive processes underlying the listening to “yes–no” questions and the answerer’s mental state and (ii) the online identification of decreased vigilance states that are detrimental (lowering performance) for BCI binary communication purposes, such as decreased alertness, drowsiness, and sleeping.

Multielectrode EEG recordings used simultaneously with the *f*NIRS system and quantitative source analysis of the different frequency bands at different sites are necessary to clarify these questions. For the study reported here, only portable devices and a few EEG channels could be used in the interest of the bedside, home-based strategy selected. Thus, our interpretation of the EEG frequency bands’ variations remains speculative.

In patients completely motionless over a period of years with restricted vision because of eye muscle paralysis and compromised vision because of drying and reduced or absent afferent input from the sensorimotor system, reduced vigilance measured with EEG and an irregular sleep–wake cycle was documented by Ramos et al. (2011) [31] and Soekadar et al. (2013) [54]. De Massari et al. (2013) [45] have shown that reduction of P300 amplitude across the BCI paradigm presentation predicted negative performance, again suggesting excessive loss and excessive variation of wakefulness and attention as a major limiting factor for BCI applications in such severely compromised patients. Thus, we modified the existing *f*NIRS–BCI–system in a hybrid EEG–*f*NIRS–BCI, with the EEG allowing online corrections of excessive reduction of vigilance indicated by appearance of delta and low-theta periods. This new hybrid system should allow further improvement of communication in CLIS.

The results on four CLIS patients reported here allow the following conclusions:

1. Even after extended CLIS in ALS spanning months and years, reliable, meaningful communication using questions requiring a mental affirmative (“yes”) or negative, rejecting (“no”) answer is possible with *f*NIRS–BCI [55,56]. This statement, however, requires a definition of “reliable and meaningful” communication between people, which is an exceedingly difficult task. For BCI spelling tasks (i.e., when participants have to select letters or words presented on a computer screen with brain activity), we [57] calculated a minimum correct selection probability of 70% for isolated selected letters to result in meaningful words over a defined time window. Anything below 70% leads to unacceptable error and correction rates. Another qualitative strategy to estimate the usefulness of the more than 70% correct answering patterns achieved here consists of the ratings of family members and caretakers—which we did not measure quantitatively—regarding quality of life changes with the BCI described here compared to the desperate lack of communication on patients’ and caretakers’ family side before BCI use. Family members of all four patients’ experienced substantial relief and continue to use the system. It seems that patients and families internally develop a seven correct to three false ratio “running average significance tests” over weeks and months, and if doubts about correctness become obvious (i.e., if the patient changes answer direction [affirmative-negative] of a repeated identical question within 2 to 3 d from 7:3 ratio to 5:5), questions are reformulated. As one can deduct from the concordance percentage of semantically paired “yes” and “no” questions, the answers were concordant in most of the cases (“Paris is the capital of France”—“yes”; “Paris is the capital of Germany”—“no.”). As, for example, with children, we and the family members and caretakers accept a higher error rate in CLIS patients than in healthy adults because of their fragile vigilance and unpredictable circadian rhythms that result in spontaneous sleep and dozing during the day [54]. Because each question has a semantically identical but contradictory answering twin question (“Berlin is the capital of Germany,” “Berlin is the capital of France”), judgement of correct answering patterns is further improved. Our result of a significant positive concordance between semantically contradictory sentences, however, supports the notion that patients processed these sentences correctly. Still, we have to remain cautious about our judgements to open questions’ answers, particularly if it comes to quality of life and psychological changes of CLIS patients. In view of the gravity of the subject matter (i.e., establishing communication with nonverbal, completely paralyzed persons with preserved cognition), a call for replication of the current results by other investigators would be welcome. Future BCI-based communication has to focus on quantitative assessment of stability (reliability) of the found positive quality of life ratings and subjective emotional states. In the above-reported patients, all questions were repeated several times over weeks of BCI used with remarkable stability of correct answering patterns, but a quantitative approach to measure reliability and stability over longer time period is desirable. Despite our theoretical predictions of the CLIS for goal-directed thinking and intentions described above in the introduction, we should never abandon our attempts to return to instrumental learning and voluntary free spelling with the help of BCI systems.
2. *f*NIRS seems to provide better classification of patients’ answers compared to oscillatory EEG responses. The above statement of a superiority of *f*NIRS over EEG–BCI needs a word of caution. The EEG oscillations were analyzed using average power over the 15 s answering period, neglecting the temporal dynamics of the EEG across the answering period. Thus, any difference in the beta and/or gamma frequency range (less so in the low frequencies) that may occur at different time points of the answering period is ignored with this type of averaging. Replications of the comparisons reported here between *f*NIRS–BCI and EEG–BCI in CLIS should employ a more complex time-frequency analysis of the EEG signals during the course of the answering period. This kind of EEG temporal dynamics analysis should investigate, at the single-trial level, relevant frequency changes at different time delays of the mental and neurophysiological signatures of the answer. With the limited number of EEG channels and the employed bandpass filter because of the home-based BCI limitations, the covert nature of the dynamics of the mental answer, and the obvious pathology of the EEG in these patients, we had to abstain from further complex analysis. In the present study, only a preliminary EEG temporal dynamics analysis based on averaged data of each session for each patient was viable (see Methods section of S1 Text). The results from two patients (F and W) partially confirm the hypothesis of superiority of *f*NIRS over EEG in the detection of true and false neurophysiological responses to “yes” and “no” sentences (see S1 Text, paragraph EEG time-frequency and *f*NIRS classification comparison). However, because the time-frequency analysis was performed at session level (i.e., on averaged data, not on single-trial data), caution is necessary in the interpretation of the results. Similar difficulties encountered using different techniques are described in a previous study of patient F and two LIS ALS patients (De Massari et al. 2013), albeit a slightly different semantic conditioning paradigm employing electrical stimulation was used. Compared to *f*NIRS, the EEG time-frequency analysis may identify specific neuroelectric frequencies’ oscillations at different time points with fine resolutions and with potential further insights in neurophysiological mechanisms underlying the engaged mental processes. Conversely, *f*NIRS signals may be more easily detected for binary classification. We have argued previously [14] the speculation that metabolic (vascular) brain changes permit superior learned brain self-control in *f*MRI neurofeedback experiments because of an existing feedback pathway between the vascular system in the central nervous system. While neuroelectric changes lack receptors systems of their own activity, the vascular bed provides accurate information of flow and diameter changes to the neuronal assemblies in its neighborhood. This allows adjustment to metabolic and cognitive needs and probably superior access to voluntary control [58], as required in the paradigm reported here: patients had to control the correct timing of their “yes” or “no” answer, otherwise correct classification of the correlated physiological signal (oxygenation) would not be possible. A physiological system such as the vascularity of the brain measured with *f*MRI and *f*NIRS provides feedback to the brain about its state changes, while the neuronal neuroelectric changes may not be “perceived” by the brain and thus provide no feedback of its present state or state changes; thus, a physiological system should be superior for instrumental learning. To put it more colloquially: physiological feedback of our thoughts (“perceiving thoughts”) is encoded in the neuronal control structures of the brain through the vascular systems and not through neuromagnetic changes such as cellular membrane polarization changes and changes in neuroplastic synapses. While thoughts probably consist of neuroelectric changes and their underlying cellular polarization across the cell membranes, their physiological consequences or correlates may appear as metabolic. Thus, coregistration of *f*NIRS and EEG and other neuroelectric changes and oscillations from multiple sites maybe important in CLIS in order to monitor and eventually modify nonfavorable vigilance changes reflected in the EEG, with arousal stimulating activities to improve NIRS classification.

## Materials and Methods

The Internal Review Board of the medical faculty of the University of Tubingen approved the experiment reported in this study, and the patients’ legal representative gave informed consent for the study with permission to publish the results and show the face of patients in the publication. The study was in full compliance with the ethical practice of medical faculty of the University of Tubingen. The clinical trial registration number is ClinicalTrials.gov Identifier: NCT02980380. At the time of this study, prospective clinical trial registration was not mandatory for nonpharmacological studies; it was therefore registered retrospectively.

### Instrumentation

A continuous wave (CW)-based *f*NIRS system, NIRSPORT (NIRX), which performs dual-wavelength (760 nm and 850 nm) CW near-infrared spectroscopic measurement at a sampling rate of 6.25 Hz, as shown in in Fig 6A, was used. The NIRS optodes were placed on the frontocentral regions as shown in Fig 6B. During the BCI sessions, the EEG was also recorded with a multichannel EEG amplifier (Brain Amp DC, Brain Products, Germany) from ten Ag/AgCl passive electrodes mounted on the head cap. Six electrodes (FC5, FC1, FC6, CP5, CP1, and CP6) were used to acquire EEG signals and four electrodes were used to acquire the vertical and horizontal EOGs. The signals were bandpass filtered using a finite impulse response filter with a bandpass of 0.5–30 Hz. The EOG was filtered with different bandpass filters (0.5–3.5 Hz, 0.5–10 Hz, and 0.5–30 Hz), but none of these filters led to significant differences of neurophysiological patterns related to the ocular activity. Question- or response-related eye movements were not detected in any of the patients over the whole time period of many weeks. Each EEG channel was referenced to an electrode on the right mastoid and grounded to the electrode placed at Fz location of the scalp. Electrode impedances were kept below 10 kΩ and the EEG signal was sampled at 500 Hz. During all BCI sessions, the spontaneous EEG was visually controlled by one of the authors (NB or BX) to avoid longer periods of slow-wave sleep during the BCI evaluation. A BCI session was initiated only if the EEG was free of high-amplitude slow activity below 4 Hz.

**Fig 6:** The procedure and flow diagram of the brain–computer interface (BCI) for communication in ALS patients. (A) The continuous wave-based portable NIRX NIRSport instrument. The device consists of eight near-infrared light sources (highlighted in red), eight detectors (highlighted in green), and the NIRS data acquisition hardware is highlighted in yellow. (B) Depicts the placement of sources and detectors (optodes) on the frontocentral region of the scalp (blue). Four sources (highlighted in red) and four detectors (highlighted in green) were placed on each hemisphere to form a channel.

### Patients

Patient F (female, 68 y old, completely locked-in state) was diagnosed with bulbar sporadic ALS in May 2007, was diagnosed as locked-in in 2009, and was diagnosed as completely locked-in May 2010, based on the diagnoses of experienced neurologists. She has been artificially ventilated since September 2007, fed through a percutaneous endoscopic gastrostomy tube since October 2007, and is in home care. No communication with eye movements, other muscles, or assistive communication devices was possible since 2010. Further details of this patient are described in Gallegos-Ayala et al. (2014) [30].

Patient G (female, 76 y old, CLIS) was diagnosed with bulbar ALS in 2010. She lost speech and capability to walk by 2011. She has been fed through a percutaneous endoscopic gastrostomy tube since September 2011, artificially ventilated since March 2012, and is in home care. She started using assistive communication devices employing one finger for communication in February 2013. Later, she was diagnosed with degeneration of vision because of cornea defects in September 2013. After the failure of the finger-communication device, an attempt was made to communicate using eye tracking in early 2014. She stopped communicating with the eye in August 2014, before the BCI was introduced, and an attempt was made to communicate with the subtle twitch of an eye lid, which was not reliable. The husband and caretakers declared no communication with her since August 2014.

Patient B (male, 61 y old, CLIS) was diagnosed with nonbulbar ALS in May 2011. He has been artificially ventilated since August 2011, fed through a percutaneous endoscopic gastrostomy tube since October 2011, and is in home care. He started communicating with a speech device in his throat from December 2011, which ultimately failed, and he started using the MyTobii eye-tracking device in April 2012. He was able to communicate with MyTobii until December 2013, after which the family members attempted to communicate by training him to move his eyes to the right to answer “yes” and to the left to answer “no,” but the response was variable. No communication was possible since August 2014.

Patient W (female, 24 y old, locked-in state on the verge of CLIS) was diagnosed with juvenile ALS in December 2012. She was completely paralyzed within half a year after diagnosis and has been artificially ventilated since March 2013, fed through a percutaneous endoscopic gastrostomy tube since April 2013, and is in home care. She was able to communicate with eye tracking from early 2013 to August 2014 but was unable to use the eye-tracking device after the loss of eye control in August 2014. After August 2014, family members were able to communicate with her by training her to move her eyes to the right to answer “yes” and to the left to answer “no” questions until December 2014. In January 2015, eye control was completely lost, she tried to answer yes by twitching the right corner of her mouth, that too varied considerably, and parents lost reliable communication contact.

All four patients reported in this manuscript were enrolled consecutively. Patients’ family approached us to get enrolled in the study because of the past work and public appearance of the corresponding author. Patients were never screened and excluded for this study. The only criterion for the inclusion in this study was that the patient should be in completely locked-in state (CLIS) or on the verge of CLIS, and family members could not communicate with eye movements or any other response with the patient. The CLIS state was then verified with confirmation of the attending neurologist, EOG recordings, and video recordings of the families’ failures to achieve contact with the patient.

### Experimental Procedures

The schematic depicting the experimental procedure, acquisition, and analysis of *f*NIRS and EEG data during BCI sessions is shown in Fig 6.

An auditory paradigm was employed to (a) train patients on questions with known answers, termed as training sessions; (b) give feedback on questions with known answers, termed as feedback sessions (i.e., “Your husband’s name is Joachim,” and after classification during ISI: “your answer was recognized as ‘yes’/‘no’); and (c) answer open questions, termed as open question sessions (“You have back pain”). Known questions are personal questions based on patient’s biography. For every known question with a clear “yes” answer, a semantically related question with a clear “no” answer was constructed and vice versa; for example, “You were born in Berlin” and “You were born in Paris.” Patients were asked to think “yes” or “no” answers and, if possible, also to use their previously successful eye movements. They were explicitly instructed not to imagine the answer or visually or auditorily imagine the word (i.e., as a visual or sound form) “yes” or “no”. Open questions are general questions related to quality of life and questions of caretakers whose answers can only be known by the patient. A total of at least 200 known questions and 40 open questions were constructed for each patient with family members before the initiation of the BCI study. Each patient was visited for 4 to 5 d in a month, except patient W. Three to four sessions were performed each day depending upon the health condition reported by the caretakers of the patient. Every session lasted for 9 min, and a session in progress was terminated extremely rarely (i.e., if removal of saliva became urgent). In such a rare event, the session was started again. Since each session lasted for 9 min, the caretaker or the family member was always instructed to take care of the needs of the patient before the start of the session, and the session was always started with the permission of the caretaker or the family member. A session, once in progress, was never terminated for patients F, G, and W. For patient B, a session was terminated while in progress three times because of removal of saliva, and the data were not included in any kind of analysis.

Acoustically presented instructions about the procedure were given repetitively before each training, feedback, and open questions sessions, allowing patients to recall and consolidate the required task to listen and answer mentally. Each BCI session started with training sessions, during which the patients were instructed to listen to 20 personal questions (with known answers) consisting of 10 true and 10 semantically equivalent false sentences. The sentences were presented randomly in such a way that two semantically related questions never played one after another. Family members were always present throughout the BCI session, and they never prompted the patient to answer the question. Complete pin-drop silence was maintained during the session, and only the recorded sentences were presented via audio presentation software connected to sound box with the voice of a family member or caregiver. Patients were asked to think “ja, ja…” (German for “yes”) and “nein, nein…” (German for “no”) for 15 s during the ISI until they heard the next sentence after an interval of 5 s of rest, as shown in Fig 6. After the end of each session, the *f*NIRS feature necessary to differentiate between “yes” and “no” answers during ISI was extracted and classified. Only training sessions were performed during the first few days, and upon several successful training sessions (as described below in BCI effectiveness metric section), the online feedback session was performed. During training sessions, both the patient and the algorithm were trained. Patients learned to mentally answer the question, and the algorithm learned to classify the “yes” and “no” *f*NIRS pattern of a particular patient. This kind of “mutual learning” seems important to optimize the “yes” versus “no” classification outcome and to customize and/or adapt the BCI system to each individual patient. At the end of each training session with 20 sentences (questions), patients were told the average classification accuracy of the session (calculated using the SVM classifier) to motivate and help patients in learning. In the course of an online feedback session, patients were presented the known questions as described above, but now at the end of the 15 s ISI they were given auditory feedback of accuracy, during which the computer said, “Your answer was recognized as yes” or “Your answer was recognized as no” depending upon the question (all sessions were videotaped and are available on request). Feedback to strengthen the conditioned response was provided only if the classification accuracy was greater than the chance-level upper limit to guide the conditioned learning toward meaningful answers and to avoid frustration by negative feedback already at the beginning of a daily session. Feedback was driven by the *f*NIRS classifier, calculated using the data acquired during the training sessions. After successful training and feedback sessions, the patients were presented with open questions, during which they were always given the auditory feedback of their answer.

The validity of answers to open questions can only be estimated by (a) face validity (i.e., questions of pain in the presence of an open wound); (b) stability over time; (c) external validity, estimated by family members and caretakers; and (d) internal validity between questions (i.e., the concordance between the answer to “I love to live” with the answer to “I rarely feel sad” [presented to all patients—except W—regularly]). Table 1, rows A, B, and C enumerate the total number of training, feedback, and open questions sessions performed by each patient, respectively. Patient W received no open questions because of low classification accuracy, which we and the parents attributed to her emotional state distracting her from concentrating on the responses because of the short time period of adaptation to the CLIS.

### BCI Effectiveness Metric

The binary BCI system effectiveness and robustness depends on its capability of correctly classifying the neurophysiological correlates of “yes” and “no” answers to true and false questions. The proposed true and false questions have two possible outcomes only, which are equally distributed with a probability of 0.5. To ensure that the classification of “yes” and “no” answers is not at chance-level, a reliable metric has to be used. Based on binomial distribution theoretical background, Müller-Putz et al. [59] defined a metric for experimental procedures with a binary outcome and multiple repetitions to determine the chance-level threshold above which the classification accuracy results can be considered as not resulting from chance. Because type and number of questions (personal questions with known answers and open questions) are partly different over days (i.e., the experimental conditions were different) the chance-level threshold was calculated on a daily basis. The daily-based chance level was computed using the formulas described in Müller-Putz et al. [59] and by taking into account the number of true and false sentences presented in a single day to each patient.

### Online Data Analysis

The *f*NIRS data was acquired online throughout all the sessions, namely training, online feedback, and open question sessions. The *f*NIRS data acquired online was normalized, filtered using different bandpass filters (0.0016–0.3), (0.01–0.3) and (0.02–0.3) and processed using modified Beer–Lambert law [60,61] to calculate the relative change in concentration of oxyhemoglobin (O_2_Hb) and deoxyhemoglobin (RHb). The choice of bandpass filter had no effect on the waveforms of signal. The relative change in O_2_Hb computed online during each session was used to train a SVM classifier model. The mean of relative change in O_2_Hb across each channel was used as a feature to train the SVM model through a 5-fold cross-validation procedure. In this study, only the relative change in O_2_Hb was used, as after the end of sessions with known answers it was observed that O_2_Hb provided stable and higher cross-validation classification accuracy than RHb. In an invasive animal study with nonhuman primates, we have also measured a superior covariation of oxygenation changes compared to deoxygenation, with intracortically recorded neural activity [49] supporting this clinical observation. Since the classification accuracy achieved was higher for O_2_Hb, the SVM model generated using O_2_Hb was used to provide online feedback for known as well as open questions sessions. If the classification accuracies for at least three consecutive “training” sessions with questions with known answers were greater than the chance-level threshold, a new model was generated using the relative change in O_2_Hb across three training sessions to give online feedback. During an online feedback session, *f*NIRS data acquired online corresponding to each ISI was processed to obtain the relative change in O_2_Hb, as described above, across all the channels. The mean of the relative change in O_2_Hb across all the channels was used as test feature to map onto model space. Upon mapping of this test feature onto the model space, the SVM predicted (called predict label) the side of the hyperplane the test feature fell on. Depending on the value of the predict label, appropriate feedback was provided to the patient: if the predict label was 0, the patient was given feedback that his or her answer was recognized as “no,” and if the predict label was 1, the patient was given feedback that his or her answer was recognized as “yes.”

### Offline Data Analysis

*f*NIRS provides three different signals: oxyhemoglobin (O_2_Hb), deoxyhemoglobin (RHb) and total hemoglobin (THb) [60,61]. As mentioned in the section Online data analysis, since the classification accuracy achieved was higher for O_2_Hb, only the results from the offline processing of O_2_Hb data will be shown along with the EEG and EOG data. The relative change in O_2_Hb, EEG, and EOG data were processed offline to determine:

a) The statistical difference in the particular physiological signal (O_2_Hb, EEG, and EOG) during the ISI of true (yes) and false (no) sentences (in the time domain).

To ascertain the difference between the averaged ISI of true and false sentences, *t*-tests were performed. *t*-test was performed separately for O_2_Hb, EEG, and EOG signals acquired from all the sessions and across all the channels in a session, averaged over many sessions varying slightly between patients. Furthermore, *t*-tests were also performed for each session between the ISI of all the ten true sentences and all the ten false sentences (“Berlin is the capital of France,” “Berlin is the capital of Germany”) across different channels in a session.

b) The statistical difference in the offline classification accuracy of the relative change in O_2_Hb, the EOG signal, and the EEG signal power spectrum during ISI corresponding to true and false sentences.

For the EEG, frequencies between 0 and 30 Hz, estimated by Welch’s method [62], were used for classification and statistical testing. ANOVA and post hoc *t*-test were used.

c) The statistical difference of frequency bands’ (i.e., delta 0.25–3.5Hz, low-theta 3.5–5Hz, high-theta 5–8Hz, low-alpha 8–10Hz, and high-alpha 10–13Hz) features averaged daily-wise from EEG signals and their relationships with *f*NIRS SVM classification accuracy.

Frequency bands’ mean power and their “variability” were estimated using Welch’s method [44,58]. For each patient, middle-frequency bands’ (i.e., high-theta, low-alpha, and high-alpha) features of “true/yes” and “false/no” sentences’ ISI were compared, as well as middle-frequency bands’ features of sentence presentation and interstimulus intervals. Successively, the averaged correlation between each low-frequency band (i.e., delta, low-theta, and high-theta) mean power and *f*NIRS classification accuracy was computed to find relevant relationships of low EEG rhythms with the BCI experimental procedure outcome. Details are provided in the Methods section of S1 Text.

### Performance of SVM Classifier

The performance of the binary SVM classifier was ascertained by plotting the ROC curve. The ROC curve was created by plotting the TPR against the FPR (obtained from the contingency table created for each session) and the average of all the sessions, separately for each patient, using the four possible outcomes of a binary SVM classifier. The formation of contingency table for training and feedback sessions for each participant is described in the Receiver operating characteristic curve section of S2 Text. Further chi-square test was performed to determine the statistical significance of the observed outcomes in the contingency table, also described in the Receiver operating characteristic curve section of S2 Text.

### Semantic Concordance Rate (SCR)

Semantic concordance rate (SCR) was calculated to ascertain the consistency and/or concordance of the answers between semantically equivalent but contrasting true and false sentences requiring “yes” and “no” answers, respectively. SCR (i.e., the percentage of concordant answers over pairs’ repetition) was calculated for all semantically related sentences presented to each patient. The method employed to calculate the semantic concordance rate is described in the Semantic concordance rate (SCR) section of S2 Text. This measure also provides indirect information about the intact cognitive processing of the presented sentences in a CLIS patient.

## Supporting Information

S1 TREND Checklist (PDF)

S1 Text EEG frequency domain analysis. (DOCX)

S2 Text Receiver operating characteristic curve and semantic concordance rate. (DOCX)

S1 Table **Section A**. Lists the daily-wise EEG frequency domain results of each patient. The number of days for each patient were: F, 14; G, 17; B, 12; and W, 6. Middle-frequency bands’ mean power and their “variability” were compared between sentence presentation interval and sentence’s ISI. See S1 Text, section Methods, paragraph EEG middle-frequency bands comparison for details. “ISI” stands for interstimuli interval. “SP” stands for sentence presentation interval. The symbol ≈ means that the null hypothesis cannot be rejected (there were no main effects of intervals or channels). The symbols < and > mean that the null hypothesis can be rejected (there was always a main effect of intervals only). The symbol * denotes a significant *p*-value. **Section B.** Enlist the averaged correlation between daily-wise EEG frequency bands’ mean power and *f*NIRS CA for each patient. The averaged correlation was computed across selected intervals (resting before session, sentence presentation, and sentence’s ISI, specified in column 3) and across all electrodes. Column 4 lists the mean and standard deviation of each averaged correlation across intervals and electrodes with CA. Column 5 lists the *p*-values of the tested null hypothesis of whether the median of averaged correlation was zero. Further, the number of days of each patient was split in successful and unsuccessful days using the chance-level threshold. Then, the hypothesis of whether the particular band mean power distribution medians of successful and unsuccessful days differed was tested (corresponding *p*-values are listed in column 6). The effect of this comparison (i.e., whether or not the second hypothesis was rejected) is reported in column 7. “Rest” stands for resting interval before sessions. “ISI” stands for interstimuli interval. “SP” stands for sentence presentation interval. “Succ.” and “Unsucc.” stand for successful and unsuccessful days, respectively. The symbol ≈ means that the band mean power medians of successful and unsuccessful days were similar. The symbol < means that the band mean power medians of successful and unsuccessful days differed significantly. The symbol * denotes a significant *p*-value. See S1 Text, section Methods, paragraph EEG low-frequency bands correlation with *f*NIRS classification accuracy for details. S1 Table data is located at https://doi.org/10.5281/zenodo.191929.
(XLSX)

S2 Table CWT and STFT true versus false recognition accuracies: the *t*-test was used to compare CWT and STFT recognition accuracies with mean *f*NIRS classification accuracy. S2 Table data is located at https://doi.org/10.5281/zenodo.192128.
(XLSX)

S3 Table Contingency table. (XLSX)

S4 Table Patient F. Contingency table formed using the average of all the training sessions. S4 Table data is located at https://doi.org/10.5281/zenodo.192398.
(XLSX)

S5 Table Patient F. Contingency table formed using the average of all the feedback sessions. S5 Table data is located at https://doi.org/10.5281/zenodo.192400.
(XLSX)

S6 Table Patient G. Contingency table formed using the average of all the training sessions. S6 Table data is located at https://doi.org/10.5281/zenodo.192401.
(XLSX)

S7 Table Patient G. Contingency table formed using the average of all the feedback sessions. S7 Table data is located at https://doi.org/10.5281/zenodo.192402.
(XLSX)

S8 Table Patient B. Contingency table formed using the average of all the training sessions. S8 Table data is located at https://doi.org/10.5281/zenodo.192406.
(XLSX)

S9 Table Patient B. Contingency table formed using the average of all the feedback sessions. S9 Table data is located at https://doi.org/10.5281/zenodo.192407.
(XLSX)

S10 Table Patient W. Contingency table formed using the average of all the training sessions. S10 Table data is located at https://doi.org/10.5281/zenodo.192408.
(XLSX)

S11 Table Patient W. Contingency table formed using the average of all the feedback sessions. S11 Table data is located at https://doi.org/10.5281/zenodo.192409.
(XLSX)

S12 Table Semantic concordance rate (the *p*-values refer to the Wilcoxon signed rank test). S12 Table data is located at https://doi.org/10.5281/zenodo.191982.
(XLSX)

S1 Fig **A. Power spectrum density.** Power spectrum density (PSD) of electroencephalographic (EEG) signal corresponding to **YES** (red solid trace) and **NO** (blue dashed trace) sentences’ ISI acquired from channel FC6 in patients **F, G, B,** and **W**. In each subplot, the *x*-axis is frequency in hertz and the *y*-axis is channel FC6 EEG in dB (μV^2^/Hz). S1A Fig data is located at https://doi.org/10.5281/zenodo.192386; https://doi.org/10.5281/zenodo.192388; https://doi.org/10.5281/zenodo.192390; https://doi.org/10.5281/zenodo.192391. **B. Electrooculogram signal.** The electrooculogram (EOG) signal corresponding to **YES** (red solid trace) and **NO** (blue dashed trace) sentences’ ISI in patients **F, G, B,** and **W**. In each subplot, the *x*-axis is time in seconds and the *y*-axis is EOG in micro volt (μV). S1B Fig data is located at https://doi.org/10.5281/zenodo.192386; https://doi.org/10.5281/zenodo.192388; https://doi.org/10.5281/zenodo.192390; https://doi.org/10.5281/zenodo.192391.
(EPS)

S2 Fig Patient F. **Receiver operating characteristic (ROC) curve of the binary support vector machine (SVM) classifier.** (A) Training and (B) feedback sessions. Each circle in the ROC curve space represents false positive rate (FPR) versus true positive rate (TPR) for each session. Sessions with the same coordinate points in the ROC space are represented by concentric circles. The red star along with the coordinate points in the ROC space represent FPR versus TPR of all the sessions combined. In the figure panels A and B, the *x*-axis is the FPR and the *y*-axis is TPR. The thick diagonal line dividing the ROC space represents chance level. Points above the diagonal represent good classification results (better than random); points below the line represent poor classification results (worse than random). S2 Fig data is located at https://doi.org/10.5281/zenodo.192398; https://doi.org/10.5281/zenodo.192400.
(EPS)

S3 Fig Patient G. **Receiver operating characteristic (ROC) curve of the binary support vector machine (SVM) classifier.** The description of this figure is the same as described in S2 Fig. S3 Fig data is located at https://doi.org/10.5281/zenodo.192401; https://doi.org/10.5281/zenodo.192402.
(EPS)

S4 Fig Patient B. **Receiver operating characteristic (ROC) curve of the binary support vector machine (SVM) classifier.** The description of this figure is the same as described in S2 Fig. S4 Fig data is located at, https://doi.org/10.5281/zenodo.192406; https://doi.org/10.5281/zenodo.192407.
(EPS)

S5 Fig Patient W. **Receiver operating characteristic (ROC) curve of the binary support vector machine (SVM) classifier.** The description of this figure is the same as described in S2 Fig. S5 Fig data is located at https://doi.org/10.5281/zenodo.192408; https://doi.org/10.5281/zenodo.192409.
(EPS)

## Abbreviations

ALS: amyotrophic lateral sclerosis
BCI: brain–computer interface
CA: classification accuracy
CLIS: complete locked-in state
ECoG: electrocorticogram
EEG: electroencephalogram
EOG: electrooculogram
ERD: event-related desynchronization
ERP: event-related brain potential
*f*MRI: functional magnetic resonance imaging
*f*NIRS: functional near-infrared spectroscopy
FPR: false positive rate
ISI: interstimuli interval
LIS: locked-in state
ROC: receiver operating characteristic
SCP: slow cortical potential
SCR: semantic concordance rate
SMR: sensory motor rhythm
SVM: support vector machine
TPR: true positive rate
